# Optimal Modeling of Anti-Breast Cancer Candidate Drugs Based on Graph Model Feature Selection

**DOI:** 10.1155/2022/8418048

**Published:** 2022-08-30

**Authors:** Rongyuan Chen, Zhixiong He, Shaonian Huang, Lizhi Shen, Xiancheng Zhou

**Affiliations:** ^1^Key Laboratory of Hunan Province for Statistical Learning and Intelligent Computation, Hunan University of Technology and Business, Hunan Changsha 410205, China; ^2^Hunan University of Technology and Business, Hunan Changsha 410205, China

## Abstract

Breast cancer is one of the most widespread and fatal cancers in women. At present, anticancer drug-inhibiting estrogen receptor *α* subtype (ER*α*) can greatly improve the cure rate for breast cancer patients, so the research and development of this kind of drugs are very urgent. In this paper, the problem of how to screen excellent anticancer drugs is abstracted as an optimization problem. Firstly, the graph model is used to extract low-dimensional features with strong distinguishing and describing ability according to various attributes of candidate compounds, and then, kernel functions are used to map these features to high-dimensional space. Then, the quantitative analysis model of ER*α* biological activity and the classification model based on ADMET properties of the support vector machine are constructed. Finally, sequential least square programming (SLSQP) is utilized to solve the ER*α* biological activity model. The experimental results show that for anticancer data sets, compared with principal component analysis (PCA), the error rate of the graph model constructed in this paper is reduced by 6.4%, 15%, and 7.8% on mean absolute error (MAE), mean squared error (MSE), and root mean square error (RMSE), respectively. In terms of classification prediction, compared with principal component analysis (PCA), the recall and precision rates of this method are enhanced by 19.5% and 12.41%, respectively. Finally, the optimal biological activity value (IC50_nM) 34.6 and inhibitory biological activity value (pIC50) 7.46 were obtained.

## 1. Introduction

In countries all over the world, the proportion of cancer in many factors harmful to people's health is increasing year by year. Breast cancer has been the most common cancer, with a mortality rate of 11.5% to 28.4% [1]. At present, in the process of studying the treatment of breast cancer, some scholars have found that an estrogen receptor *α* subtype (estrogen receptor alpha, ER*α*) can be used as a key target for effective treatment of breast cancer, and compounds that can antagonize the activity of ER*α* can be used as candidate drugs for the treatment of breast cancer.

There are many kinds of anticancer compounds, and the extraction of low-dimensional features with strong description ability from various properties of the compounds can greatly improve the efficiency of screening anticancer drug candidates. Many scholars' abstract anticancer drug selection as feature extraction, such as Tassenberg et al. [2], use automatic feature extraction algorithm DenMap to detect single crystal dendrite core quickly, accurately, and repeatably and realize average automated feature extraction. Xue et al. [3] adopted an analytic hierarchy process entropy (HDE) feature extraction method based on the analytic hierarchy process to effectively diagnose the fault of rolling bearings, which eliminates the redundant information between features and retains the fault-related information. Yang et al. [4] used nonlinear simulation feature extraction to complete the tasks of speech detection and keyword location in inference sensor system with low power consumption. Xue et al. [5] proposed a feature extraction method based on asymmetric probability distribution function to reconstruct the distillation curve in industrial refining process, which is beneficial to the modeling and optimization of the oil refining process. Liu et al. [6] used feature extraction method to classify the biogenetic mechanism of circular RNA, which confirmed the view that multiple biogenetic mechanisms of different subsets of human CircRNA coexist. Zhu et al. [7] proposed a lightweight single image superresolution network with an expectation-maximization attention mechanism (EMASRN) to extract feature maps of different sizes. The experimental results demonstrate the superiority of EMASRN over state-of-the-art lightweight SISR methods in terms of both quantitative metrics and visual quality.

On the other hand, whether anticancer compounds can be selected as drug candidates, we also need to consider the following five characteristics: (1) intestinal epithelial cell permeability, (2) cytochrome P450 enzyme, (3) cardiac safety evaluation of compounds, (4) human oral bioavailability, and (5) micronucleus test. These five characteristics are often referred to as ADMET properties [8–10].

For the evaluation of the screening of anticancer compounds listed above, this problem is abstracted as the problem of classification and prediction of anticancer drugs based on ADMET properties. For example, Guo et al. [11] proposed a novel Relation Separation Network (RSNet) in this paper, aiming to boost few-shot learning by improving similar-class recognition performance. Compared to PT+MAP, RSNet improves the accuracy of classification on the CUB data set by approximately 5% and that of similar-class classification by more than 10%. Wang et al. [12] used a scalable window waveform sampling method (SWWS) based on the classification pattern to classify the workload requested by all users and then reasonably predict the usage of user cloud resources to minimize the cost of use. Wang et al. [13] combined missing value analysis with likelihood ratio test, introduced weighted decay random forest model, realized ICU readmission classification based on sparse data, and greatly reduced patients' expenses. Zhang et al. [14] adopted recursive partition classification method, established a classification prediction model of 58 between derivative inhibitors and du's amastigotes, and determined its molecular target and molecular mechanism. Steckenrider and Furukawa [15] adopted a highly random road crack perception network detection and classification method based on probability formula, which allows features to be extracted from crack images and retains the uncertainty in the detection. Chen et al. [16] adopted a classification diagnosis method combining FTIR near-infrared spectroscopy (NIRS) and support vector machine to differentiate malignant pleural effusion (MPE) from benign pleural effusion (BPE). Barth et al. [17] adopted the classification method of combining principal component analysis (PCA) with *K*-nearest neighbor (KNN) to address the problem of high correlation variables in wine classification. Lamge et al. [18] adopted a skin disease detection and classification method based on the combination of image processing technology and neural network to classify and evaluate patients' skin lesions images. Schultz et al. [19] used recurrent neural network and convolution neural network to classify airport performance on the basis of weather data. This method quantifies the correlation between airport performance decline and weather severity, and the prediction accuracy of aircraft take-off can reach more than 90%.

At present, the research and development of anticancer compounds in the medical field can be roughly classified into three steps. Firstly, the properties of the compounds were examined, and then, the activity model of the compound against cancer cells and the classification model of ADMET properties were constructed. Finally, the characteristic value of the antagonistic activity of the compound to cancer cells was obtained by solving the model. Therefore, in this paper, the research and development of anti-breast cancer drugs are abstracted as an optimization problem, and an optimization method based on graph model feature extraction is constructed. In this paper, the kernel function is used to map the features to a higher dimensional space to construct a nonlinear quantitative prediction function of biological activity, and then, a classification prediction model of ADMET properties of anticancer drugs based on support vector machine (SVM) is constructed as a constraint. Sequential least square programming (SLSQP) is used to efficiently and quickly solve the distinguishing variable value of the optimal biological activity value, the optimal biological activity value (IC50_nM), and the inhibitory biological activity value (pIC50). Specifically, we have studied the following four specific issues:

- Question 1: For a wide variety of compounds, can the graph model method designed in this paper extract low-dimensional features with stronger description ability from many attributes than the principal cost analysis method?
- Question 2: Can the quantitative prediction model constructed by regression method accurately predict the biological activity of ER*α*?
- Question 3: Compared with principal component analysis, can support vector machine predict ADMET properties more accurately in a shorter time?
- Question 4: Can the improved sequential least square programming (SLSQP) be solved faster and more accurately than the traditional intelligent optimization algorithm?

Through the research to solve the above problems, we can efficiently and intelligently predict whether the compound can become a candidate for breast cancer treatment and assist human doctors to accurately select effective anti-breast cancer drugs for breast cancer patients. Effectively improve the cure rate of breast cancer. The specific contributions of this article are as follows:

1. A graph model method is proposed to extract low-dimensional features with strong descriptive ability and eliminate redundant features
2. Through the graph model-SVM classification prediction method, five classification models for the properties of ADMET are constructed to test whether the candidate drugs are suitable for patients
3. The bioactivity function of anticancer drug ER*α* was constructed, and the candidate anticancer drug ER*α* with optimal bioactivity was obtained by SLSQ algorithm as the best anticancer drug

## 2. Overview of Methods

The purpose of this paper is to select candidate drugs with superior efficacy from many anti-breast cancer compounds. First of all, the low-dimensional features with strong ability to describe effectively are selected from the many attributes of the compound. Then, the activity of the compound against cancer cells is measured to determine whether the compound can be used as a candidate drug. Below, we will describe the methodology framework and technical details in detail.

### 2.1. General Framework

The overall framework of this approach is shown in Figure 1. The steps for screening anticancer drugs are as follows:

- Step 1: use the graph model method to extract low-dimensional features with strong distinguishing ability from anti-breast cancer drug candidates
- Step 2: the kernel function is used to map the extracted features to high-dimensional space to construct a quantitative analysis model of ER*α* biological activity
- Step 3: at the same time, anti-breast cancer drugs also need to consider the properties of ADMET, using SVM to build a classification prediction model
- Step 4: taking the ER*α* biological activity function in step 2 as the objective function and the classification prediction model in step 3 as the constraint, the improved least square method-sequential least square programming (SLSQP) is used to solve the optimal ER*α* biological activity value

### 2.2. Graph Model-Minimum Spanning Tree (MST)

In view of the large number of attributes of anticancer drugs, we compare the attributes of compounds to nodes in graph theory and the correlation between attributes to the distance between nodes, from which the adjacency matrix between attributes is established. Finally, all nodes can generate a minimum spanning tree to extract low-dimensional features with strong description ability. When constructing the adjacency matrix, we need to choose an appropriate threshold to construct the adjacency matrix, so the crux of the problem is how to select the applicable threshold.

First of all, *N* characteristic attributes of anticancer drugs are expressed as follows:

(1) $$\begin{array}{c} T^{0}=\left\{T_{m,n}^{O},m=1,2,\cdots ,M;n=1,2\cdots ,N\right\}, \end{array}$$

where *T*_*m*,*n*_^*O*^ is the data of the *n*(th) feature in the *m*(th) sample and *N* = 729, *M* is the number of samples. The correlation coefficient matrix is

(2) $$\begin{array}{c} R_{n_{1,}n_{2}}=\frac{\sum_{m=1}^{M}\left[T_{n_{1},m}-\left(T_{n_{1}}\right)\right]\times \left[T_{n_{2},m}-\left(T_{n_{2}}\right)\right]}{\sqrt{\sum_{m=1}^{M}{\left[T_{n_{1},m}-\left(T_{n_{1}}\right)\right]}^{2}}\sum_{m=1}^{M}{\left[T_{n_{2},m}-\left(T_{n_{2}}\right)\right]}^{2}}, \end{array}$$

where *T*_*n*_1_,_*T*_*n*_2_,_are the two features of*n*_1_, *n*_2_(th) and the similarity degree *D* between the features is defined as follows:

(3) $$\begin{array}{c} D_{n_{1,}n_{2}}=1-\left|R_{n_{1,}n_{2}}\right|. \end{array}$$

Then, the Kruskal algorithm is used to generate the minimum spanning tree according to the distance matrix and then according to the correlation coefficient between nodes. *H*(*H* < *N*) important features (nodes) are selected. If these nodes are connected, the similarity between them is calculated, and the maximum distance value is selected as the threshold *DNI*_min_ of the adjacency matrix.

### 2.3. Support Vector Machine (SVM)

ADMET properties of anti-breast cancer compounds determine whether they can be used as candidate drugs, and the quality of the index can be regarded as a multiattribute dichotomous problem. In order to meet the requirements of Question 3, this paper takes *N* compound attributes of anticancer drugs as independent variables and ADMET properties as dependent variables and then constructs five classification prediction models, which are compared with the principal component analysis.

The attribute data dimension of anticancer compounds is quite high, and there is a lot of redundancy. If the classification algorithm is directly used for classification, it is difficult to get satisfactory results in a short time. Therefore, this paper comprehensively applies SVM algorithm and graph model to classify and predict. The model framework is shown in Figure 2. The ideas are as follows:

- For high-dimensional attribute data of compounds, the graph model is used to extract low-dimensional features with strong descriptive ability to reduce redundant information
- SVM is a good binary classifier, and satisfactory results can be obtained with fewer samples

### 2.4. Kernel Function and Sequential Least Square Programming (SLSQP)

In this paper, the low-dimensional features of compounds with strong descriptive ability are screened out by the graph model, and these features are mapped to high-dimensional space by kernel function to further strengthen the ability of differentiation. Then, the best nonlinear ER*α* bioactivity model was fitted by the least square method.

The relationship between features is nonlinear, and the least square method cannot effectively fit the nonlinear relationship, so we increase the least square algorithm. For solving nonlinear programming problems, it is of great importance whether the objective function and constraint conditions are continuous and smooth. If smooth, all decision variables are differentiable. The vector composed of partial derivatives of multivariate function can be used as the gradient direction indicating the fastest growth of empirical function. As the introduction of ADMET property increases the complexity of solving the problem, we add a Lagrange multiplier method (Lagrange multiplier) to the least square algorithm and transform the constrained optimization problem into an unconstrained problem by introducing additional variables. For this reason, we construct sequential least square programming (sequential least square programming optimization algorithm, SLSQP). SLSQP efficiently preserves the nonlinear relationship between features. When solving the parameters, this method can consider the constraints other than the objective function at the same time, which meets the need of considering the ADMET properties of anticancer compounds in Question 3. The basic description of the square programming problem is as follows:

(4) $$\begin{array}{c} \begin{array}{c} \min F\left(x\right)\\ \text{subject to }C_{j}\left(x\right)=0,\;j=1,\cdots ,MEQ\\ C_{j}\left(x\right)\geq 0,\;j=MEQ+1,\cdots ,M\\ XL\leq x\leq XU,\;I=1,\cdots ,N \end{array} \end{array}$$

In equation (4), *F*(*x*) is the objective function. *C*_*j*_(*x*) = 0 is the equality constraint. *C*_*j*_(*x*) ≥ 0 is the inequality constraint. *XL* and *XU* are the lower and upper bounds of the variable *x*. The solution process of the algorithm is as follows:

- Step 1: given the initial point *x*^0^ and convergence accuracy *ϵ*, set the parameter *k* = 0
- Step 2: *F*(*x*)  is added to the Lagrangian operator at *x*^0^ for Taylor expansion, and the current optimal solution *s*^*k*^ is calculated
- Step 3: *s*^*k*^ is taken as the search direction of the next iteration, and the next iteration point *x*^*k*^ is obtained by one-dimensional search of *F*(*x*) according to constraints
- Step 4: if *x*^*k*+1^ satisfies the termination criterion of a given accuracy, *x*^*k*+1^ is taken as the optimal solution and *F*(*x*^*k*+1^) as the optimal cost of the objective function to terminate the calculation

## 3. Experimental Results and Analysis

In this section, we introduce the experimental environment, the source of the data set, and the specific experimental results. Depending on the four research questions designed, we have carried out comparative experiments and analysis.

The program is clearly understood by Python3.6 programming, and the program runs on a microcomputer with CPU 2.40 GHz and 8 GB memory.

The data set used throughout this paper is the D problem data set provided by the 18th Huawei Cup Mathematical Modeling Competition. The data set contains a large number of 729 attribute data of anti-breast cancer compounds and the corresponding ADMET property data.

### 3.1. Question 1: Feature Selection of Anticancer Drugs Based on Graph Model

The similarity between the characteristic variables is computed according to the degree change between the minimum spanning tree nodes. The positive and negative degree changes of some of the nodes are given in Table 1. If they are greater than the threshold *DNI*_min_, the two nodes are connected, and the value is 1 in the adjacency matrix. Otherwise, the value is 0. Finally, the minimum spanning tree of all nodes is obtained, and the degrees of all nodes are calculated and arranged in a descending order. The size of the value is invoked as the additional weight of the feature.

First, standardize the integrated data; then, use the graph model to solve the weight coefficients of 729 feature components; and select the first 15 feature components according to the weight, as shown in Table 2.

In order to make a quantitative comparison with PCA algorithm, MAE (mean absolute error), MSE (mean squared error), and RMSE (root mean square error) are selected to evaluate the effect of feature extraction. Among them, MAE is the average of the absolute error which can represent the actual situation of the predicted error. MSE is the expected value of the square of the difference between the estimated value and the true value of the parameter. RMSE is the arithmetic square root of MSE. They all can evaluate the change degree of the data, and the smaller their values are, the better the accuracy of the prediction model which provides a description of the experimental data. The calculation formula of each index is as follows:

(5) $$\begin{array}{c} \text{MAE}=\frac{1}{m}\overset{m}{\underset{i=1}{\sum }}\;\left|\left(y_{i}-\hat{y_{i}}\right)\right|,\\ \text{MSE}=\frac{1}{m}\overset{m}{\underset{i=1}{\sum }}\;{\left(y_{i}-\overset{\wedge }{y_{i}}\right)}^{2},\\ \text{RMSE}=\sqrt{\frac{1}{n}\overset{n}{\underset{i=1}{\sum }}\;{\left({\overset{\wedge }{y}}_{i}-y_{i}\right)}^{2}}. \end{array}$$

The comparison of the three indicators of the algorithm and PCA for the data set of anti-breast cancer compounds is shown in Table 3.

It can be seen in Table 3 that the error index of the graph model is smaller and better than that of the principal component analysis. In MAE, the error rate of the graph model is 6.4% lower than that of PCA. In MSE, the error rate of the graph model is 15% lower than that of PCA. In RMSE, the error rate of the graph model is 7.8% lower than that of PCA. This shows the superiority of the graph model in extracting essential feature indexes and provides excellent characteristic variables for the construction of quantitative analysis model of biological activity of compounds against ER*α*.

### 3.2. Question 2: Quantitative Prediction of the Biological Activity of Anticancer Substances against ER*α*

In this paper, the kernel function is used to fit the low-dimensional features extracted from problem 1 many times by high-dimensional mapping to fit the nonlinear function. The fitting effect of the model is the best when the number of variables is 2 (for example, *x*^2^_*i*_); that is, the new 135 features can be constructed from the kernel function through 15 feature variables and compared with Adaboost regression and Lasso regression. The fitting effect diagram and model evaluation comparison table are shown in Figure 3 and Table 4.

As can be seen from Figure 3, the nonlinear function fitted by high-dimensional mapping of features by using kernel functions has a good fitting effect on the test set data, and most of the predicted data sets are consistent with the test set data. The fitting degree score of the function is 0.6231.

As can be seen from Table 4, compared with Adaboost and Lasso, the sequential least square programming constructed in this paper reduces the error rate by 22.4% and 32.2% on MAE, 23.8% and 44.3% in MSE, and 12.7% and 25.4% in RMSE and increases the fitting degree by 19.4% and 48.0%, respectively. This shows that the nonlinear inhibition ER*α* bioactivity optimization model constructed by sequential least square programming has good fitting effect and a small error.

Therefore, this paper constructs the following objective function:

(6) $$\begin{array}{c} \max F\left(x_{1},x_{2},\cdots ,x_{15}\right)=\overset{i=15}{\underset{i=1}{\sum }}k_{i}x_{i}+{\left(\overset{i=15}{\underset{i=1}{\sum }}k_{i}x_{i}\right)}^{2}+b,\;i=1,2,\cdots ,15, \end{array}$$

where *x*_*i*_ is the characteristic variable, *k*_*i*_ is the regression coefficient, and *b* is the intercept of the function. The polynomial coefficients $\hat{k_{m}}\left(m=1,2,\cdots ,135\right)$ (partial display) are shown in Table 5.

As can be seen from Table 5, the regression coefficients of these 135 features can be divided into three types: greater than 0, less than 0, and equal to 0. From the mathematical point of view, we can see that there is an inflection point in the model; that is, there is a local optimal solution. Among them, the characteristic of regression coefficient greater than 0 was positively correlated with the inhibition of cancer cell activity, the characteristic of regression coefficient less than 0 was negatively correlated with the inhibition of cancer cell activity, and the characteristic of regression coefficient equal to 0 had no effect on the inhibition of cancer cell activity.

### 3.3. Question 3: Classification Prediction Results of ADMET Properties of Anticancer Substances Based on Support Vector Machine (SVM)

Considering the high-dimensional attributes of anticancer compounds, firstly, PCA and graph model are used to extract features with strong distinguishing ability, and then, SVM algorithm is used to classify the features, and then, the optimal classification prediction model MST-SVM of compound ADMET is constructed and compared with PCA-SVM model. The operation flow chart of Question 3 is shown in Figure 4.

Based on the 15 important features extracted by the graph model, the 15-dimensional features are input into the SVM classification model combined with the compound ADMET properties (0 or 1) for classification prediction. The classification results are shown in Figures 5–9.

Among them, blue dots and orange dots in all the classification effect maps represent 0 and 1, respectively, that is, the ADMET properties of the compound. From the classification effective images of the above five property classification models, we can see that the classification effect is obvious, and the positive and negative samples can be well distinguished. This shows that the classification prediction model of ADMET properties of MST-SVM compounds has a good classification effect. In order to make a more accurate quantitative analysis, we further introduce four indicators, namely, accuracy, accuracy, recall, and F1-score, to evaluate the classification effect, as shown in Table 6.

As can show in Table 6, the classification prediction models based on the properties of Caco-2, CYP3A4 and MN are 0.8580, 0.9379 and 1.0000 in recall, respectively. This shows that there are small false counterexamples in the classification model, and the model can achieve good results in predicting correct counterexamples. The classification prediction models based on CYP3A4 and hERG properties are 0.8947 and 0.8643 in precision, respectively. This shows that there are few correct examples in the prediction of the classification model, and the model can achieve good results in predicting the correct instances. At the same time, in accuracy, all the five classification models have higher accuracy scores. This shows that the graph model-support vector machine classification prediction model set out in the present paper can accurately judge whether the candidate drugs conform to the ADMET properties.On the basis of the above, the classification results of the ADMET properties of compounds by this method and PCA-SVM are compared as showed in Table 7:

It can be seen from Table 7 that the score of the classification prediction model of ADMET properties of PCA-SVM compounds is better than that of the MST-SVM classification prediction model in accuracy and F1-score. However, the PCA-SVM model performs poorly in the recall and precision indexes. It is worth noting that in the HOB property classification, the recall and precision of the PCA-SVM model are both 0, indicating that the stability of the model in this property classification is weak. It can be seen that the high score of accuracy in additional property classification of the PCA-SVM model cannot accurately evaluate the classification effect. On the contrary, the MST-SVM model performs well in each evaluation index, and the overall score of recall and precision is better than that of the PCA-SVM model, with an average increase of 19.5% and 12.41% in recall and precision, indicating that its classification effect is stable. Therefore, based on the above analysis, this paper chooses the MST-SVM classification prediction model which is more stable.

### 3.4. Question 4: Sequential Least Square Programming (SLSQP) Is Used to Solve the Quantitative Prediction Model of the Bioactivity of Anticancer Substances against ER*α*

In this paper, the compound is required to optimize the inhibition of ER*α* biological activity (pIC50 value) under the premise of satisfying ADMET properties (at least three properties), so that the pIC50 value is the best (the higher the better), and the corresponding characteristic variables are obtained. In this paper, the equation (6) is taken as the objective function, and 15 important characteristic variables are numerically constrained.

(7) $$\begin{array}{c} \left\{\begin{array}{c} 10\leq X_{1}\leq 50,\\ 3\leq X_{2}\leq 12,\\ 0\leq X_{3}\leq 0.00001,\\ 0.5\leq X_{4}\leq 0.7,\\ 5\leq X_{5}\leq 6.5,\\ 0.4\leq X_{6}\leq 0.6,\\ 0\leq X_{7}\leq 2,\\ -0.36\leq X_{8}\leq -0.35,\\ 0.5\leq X_{9}\leq 1,\\ 0.04\leq X_{10}\leq 0.3,\\ 0\leq X_{11}\leq 3,\\ 2\leq X_{12}\leq 3,\\ -0.1\leq X_{13}\leq -0.008,\\ 3.6\leq X_{14}\leq 15,\\ 60\leq X_{15}\leq 80. \end{array}\right. \end{array}$$

By solving the model composed of equations (6) and (7), the optimal pIC50 value is obtained. Then, the ADMET property of the compound is tested; that is to say, the SVM classification prediction model is used to make a classification prediction according to the 15 variables *x*_*i*_ to be obtained in this problem. If the variables can satisfy more than 3 ADMET properties, then the values of the variables *x*_*i*_ and pIC50 are directly output as the final optimization scheme, and if they are not satisfied, the new variable ${\dot{x}}_{i}$ is put into the constraint to judge.

The mathematical expression of ADMET property constraints is as follows:

(8) $$\begin{array}{c} M_{\text{Caco}‐2}\left\{\begin{array}{cc} 1, & \text{the property is good},\\ 0, & \text{the property is poor}, \end{array}\right.\\ M_{\text{CYP}3\text{A}4}\left\{\begin{array}{cc} 1, & \text{the property is poor},\\ 0, & \text{the property is good}, \end{array}\right.\\ M_{\text{hERG}}\left\{\begin{array}{cc} 1, & \text{the property is poor},\\ 0, & \text{the property is good}, \end{array}\right.\\ M_{\text{HOB}}\left\{\begin{array}{cc} 1, & \text{the property is good},\\ 0, & \text{the property is poor}, \end{array}\right.\\ M_{\text{MN}}\left\{\begin{array}{cc} 1, & \text{the property is poor},\\ 0, & \text{the property is good}. \end{array}\right. \end{array}$$

Finally, we obtained the optimal inhibitory activity value of ER*α* and the corresponding characteristic variable *x*_*i*_ value. The results are shown in Table 8.

Depending on the above table, under the constraint of the ADMET property of the compound, the values of 15 characteristic variables, the optimal bioactivity value (IC50_nM), and the inhibitory bioactivity value (pIC50) were obtained. Among them, the distinguishing variable of positive value was positively correlated with the biological activity of ER*α*. The characteristic variable of negative value was negatively correlated with the biological activity of ER*α*, and the characteristic variable of 0 value had no effect on the biological activity of ER*α*. Finally, the functional relationship between inhibitory activity value and biological activity value is presented in the following equation:

(9) $$\begin{array}{c} F_{2}=9-\log_{10}F_{1}. \end{array}$$

In equation (9), *F*_1_ is the value of biological activity and *F*_2_ is the value of inhibitory activity.

It is found that 15 characteristic variable inputs satisfy more than 3 ADMET properties when they are put into the constraint. This demonstrates that the low-dimensional features screened by the graph model not only have strong ability to describe and distinguish but also perform better through ADMET properties. It can be seen that the quantitative analysis model of ER*α* biological activity and the classification model based on ADMET properties of the support vector machine can quickly and accurately screen effective compounds from anti-breast cancer drug candidates. The running time of the experimental program is 0.1369 s, and the number of iterations is 22. From the analysis of time complexity and iterative process, sequential least square programming (SLSQP) algorithm constructed in this paper is better than the traditional intelligent optimization algorithm (such as ant colony algorithm, genetic algorithm).

## 4. Conclusions

In view of the increasing number of breast cancer patients, various kinds of anti-breast cancer candidate drugs, and great pressure on doctors to use anti-breast cancer drugs, this paper is aimed at the problem of screening anti-breast cancer candidate drugs that propose an optimal modeling method of anti-breast cancer candidate drugs based on graph model feature extraction. Compared with the traditional feature extraction methods (such as principal component analysis and random forest), the graph model feature extraction method proposed in this paper addresses the problem of large error and low accuracy of the existing methods in the evaluation index. At the same time, the classification prediction model constructed in this paper is utilized to effectively detect whether the drug will have adverse reactions to the human body when screening candidate drugs. Therefore, through the method of this paper, we can efficiently and intelligently predict whether the compound can become a candidate drug for the treatment of breast cancer and assist human doctors to accurately select effective anti-breast cancer drugs for breast cancer patients, which is of great significance to improve the cure rate of breast cancer.

## Figures and Tables

**Figure 1:** the overall framework.

**Figure 2:** Graph model framework of ADMET property classification and prediction model for SVM compounds.

**Figure 3:** Optimize the fitting effect of the model for inhibiting the biological activity of ER*α*.

**Figure 4:** Question 3 operation flow chart.

**Figure 5:** Classification effect diagram based on property Caco-2.

**Figure 6:** Classification effect diagram based on property CYP3A4.

**Figure 7:** Classification effect diagram based on property hERG.

**Figure 8:** Classification effect diagram based on property HOB.

**Figure 9:** Classification effect diagram based on property MN.

**Table 1:** The degree change of the minimum spanning tree of some feature nodes.

Features	Nodes Degree_1	Nodes Degree_0	Nodes Degree_diff	Features	Nodes Degree_1	Nodes Degree_0	Nodes Degree_diff
nHCsatu	190	23	167	MDEN-11	142	33	109
nG12Ring	156	0	156	MLFER_BH	178	69	109
SHCsatu	167	16	151	maxdNH	140	31	109
nHBint3	166	29	137	mindNH	139	31	108
ETA_Shape_Y	70	207	137	minHdNH	138	31	107
maxHBd	38	167	129	maxaasC	73	179	106
SsNH2	158	29	129	nBondsD2	211	106	105
nsNH2	158	30	128	minsCH3	31	135	104
nHsNH2	158	30	128	MDEN-12	137	33	104
SHsNH2	158	32	126	SHBint2	173	69	104
ATSm1	158	33	125	minHBd	49	151	102
SHdNH	155	31	124	nBase	162	61	101
minHCsats	12	136	124	minaaaC	43	144	101
SdNH	154	31	123	minHBint6	2	102	100
nHdNH	154	31	123	SHBint8	156	57	99
ndNH	154	31	123	SHsOH	81	180	99
ATSc5	142	20	122	nHBint2	163	66	97
nHBint7	157	37	120	SsssCH	179	82	97
nHBint8	162	46	116	SaaaC	43	139	96
MLFER_BO	179	68	111	maxsCH3	43	138	95
SHBint3	167	56	111	maxaaaC	46	141	95
ndssC	168	58	110	nsssCH	194	100	94
XLogP	73	183	110	minHsOH	68	161	93
nHBint10	165	55	110	maxssssC	96	4	92
maxHdNH	141	31	110	SdO	200	108	92

**Table 2:** Weight ranking of the first 15 feature variables in graph model extraction.

Feature number	Feature name	Weight
659	MDEC-23	0.110333
587	LipoaffinityIndex	0.100936
406	minsssN	0.075303
476	maxHsOH	0.036822
531	maxssO	0.036599
357	minHsOH	0.031988
56	C1SP2	0.025563
39	BCUTc-1 l	0.024249
673	MLFER_A	0.016138
652	MLogP	0.016063
79	VC-5	0.012582
639	nHBAcc	0.010918
351	minHBint5	0.010303
410	minsOH	0.009069
103	CrippenLogP	0.007243

**Table 3:** Error results of two feature extraction algorithms.

Arithmetic	Evaluation index		
	MAE	MSE	RMSE
Graph model	0.5217	0.5044	0.7102
PCA	0.5571	0.5936	0.7704

**Table 4:** Comparison table of model evaluation results.

Arithmetic	Evaluation index			
	MAE	MSE	RMSE	Score
SLSQP	0.6587	0.7715	0.8783	0.6231
Adaboost	0.8492	1.0127	1.0063	0.5023
Lasso	0.9721	1.3849	1.1767	0.3236

**Table 5:** Regression coefficient $\hat{k_{m}}$ result (partial display).

Regression coefficient $\hat{k_{m}}$	Regression coefficient value
$\hat{k_{1}}$	1.5541*e*-07
$\hat{k_{2}}$	-0.0029
$\hat{k_{3}}$	0.2517
$\hat{k_{4}}$	-0.0141
$\hat{k_{5}}$	0
$\hat{k_{6}}$	-0.3898
$\hat{k_{7}}$	0
$\hat{k_{8}}$	0.1859
$\hat{k_{9}}$	0
$\hat{k_{10}}$	0
$\hat{k_{11}}$	0
$\hat{k_{12}}$	0.4203
$\hat{k_{13}}$	-0.0173
$\hat{k_{14}}$	0
⋮	⋮
$\hat{k_{131}}$	-0.1225
$\hat{k_{132}}$	-0.0051
$\hat{k_{133}}$	-0.0038
$\hat{k_{134}}$	-0.0008
$\hat{k_{135}}$	0.0001

**Table 6:** Graph model-SVM various accuracy results of classified prediction models.

ADMET	Accuracy	Recall	Precision	F1-score
Caco-2	0.8127	0.8580	0.7616	0.8141
CYP3A4	0.8734	0.9379	0.8947	0.8704
hERG	0.8025	0.7713	0.8643	0.8034
HOB	0.7392	0.0381	0.6667	0.6420
MN	0.7443	1.0000	0.7443	0.6352

**Table 7:** Accuracy comparison of ADMET property classification prediction model in two classification algorithms.

	Accuracy		Recall		Precision		F1-score	
	PCA-SVM	MST-SVM	PCA-SVM	MST-SVM	PCA-SVM	MST-SVM	PCA-SVM	MST-SVM
Caco-2	0.8633	0.8127	0.9136	0.8580	0.7878	0.7916	0.8643	0.8141
CYP3A4	0.8785	0.8734	0.9000	0.9379	0.9321	0.8947	0.8802	0.8704
hERG	0.8228	0.8025	0.8430	0.7713	0.8430	0.8643	0.8228	0.8034
HOB	0.7342	0.7392	0.0000	0.7381	0.0000	0.6667	0.6212	0.6420
MN	0.7722	0.7443	0.9966	1.0000	0.7670	0.7443	0.6990	0.6352

**Table 8:** Solution results of bioactivity optimization model for inhibition of ER*α*.

Characteristic variable *x*_*i*_	MDEC-23	10
	LipoaffinityIndex	12
	minsssN	0
	maxHsOH	0.5
	maxssO	6.5
	minHsOH	0.6
	C1SP2	0
	BCUTc-1 l	-0.36
	MLFER_A	1
	VC-5	0.3
	nHBAcc	3
	minHBint5	3
	ATSc3	-0.1
	MDEC-33	12.9
	TopoPSA	80

Biological activity	IC50_nM	34.6

Inhibitory bioactivity	pIC50	7.46

## Data Availability

The data that support the findings of this study are available from the corresponding author upon reasonable request.

## References

[1] Nguyen X., Hooper M., Borlagdan J. P., Palumbo A. (2021). A review of fam-trastuzumab deruxtecan-nxki in HER2-positive breast cancer. *Annals of Pharmacotherapy*.

[2] Tassenberg K., Nenchev B., Strickland J., Perry S., Weston D. (2021). Den Map single crystal solidification structure feature extraction: automation and application. *Materials Characterization*.

[3] Xue Q., Xu B., He C. (2021). Feature extraction using hierarchical dispersion entropy for rolling bearing fault diagnosis. *IEEE Transactions on Instrumentation and Measurement*.

[4] Yang M., Liu H., Shan W. (2021). Nanowatt acoustic inference sensing exploiting nonlinear analog feature extraction. *IEEE Journal of Solid-State Circuits*.

[5] Xue Y., Wang Y., Sun B. (2020). Asymmetric probability distribution function-based distillation curve reconstruction and feature extraction for industrial oil-refining processes. *Energy & Fuels*.

[6] Chengyu L., Yu-Chen L., Hsien-Da H., Wang W. (2020). Biogenesis mechanisms of circular RNA can be categorized through feature extraction of a machine learning model. *Bioinformatics*.

[7] Zhu X., Guo K., Ren S., Hu B., Hu M., Fang H. (2022). Lightweight image super-resolution with expectation-maximization attention mechanism. *IEEE Transactions on Circuits and Systems for Video Technology*.

[8] Gajjar Normi D., Dhekelia Tejas M., Shah G. B. (2021). In search of RdRp and Mpro inhibitors against SARS CoV-2: molecular docking, molecular dynamic simulations and ADMET analysis. *Journal of Molecular Structure*.

[9] Bhakhar Kaushikkumar A., Gajjar Normi D., Bodiwala Kunjan B., Sureja Dipen K., Dhameliya T. M. (2021). Identification of anti-mycobacterial agents against mmpL3: virtual screening, ADMET analysis and MD simulations. *Journal of Molecular Structure*.

[10] ElHuda D. N., Pobitra B., Kishore D. P. (2021). ADMET profiling in drug discovery and development: perspectives of in silico, in vitro and integrated approaches. *Current Drug Metabolism*.

[11] Guo K., Shen C., Hu B., Hu M., Kui X. (2022). RSNet: relation separation network for few-shot similar class recognition. *IEEE Transactions on Multimedia*.

[12] Wang X., Cao J., Yang D., Qin Z., Buyya R. (2021). Online cloud resource prediction via scalable window waveform sampling on classified workloads. *Future Generation Computer Systems*.

[13] Wang B., Ding S., Liu X., Li X., Li G. (2021). Predictive classification of ICU readmission using weight decay random forest. *Future Generation Computer Systems*.

[14] Yuezhou Z., Henri X., Leo G. (2020). Predictive classification models and targets identification for betulin derivatives as Leishmania donovani inhibitors. *Journal of Cheminformatics*.

[15] Steckenrider J., Furukawa T. Continuum detection and predictive-corrective classification of crack networks.

[16] Chen Z., Chen K., Lou Y., Zhu J., Mao W., Song Z. (2021). Machine learning applied to near-infrared spectra for clinical pleural effusion classification. *Scientific Reports*.

[17] Barth J., Catenulate D., Yang C., Cao J. (2021). Classification of wines using principal component analysis. *Economics*.

[18] Lamge R., Karmaran V., Hakke G., Pansambal S. (2020). Skin disease detection and classification using image processing algorithm. *SAMRIDDHI: A Journal of Physical Sciences, Engineering and Technology*.

[19] Schultz M., Reitmann S., Alam S. (2021). Predictive classification and understanding of weather impact on airport performance through machine learning. *Transportation Research Part C Emerging Technologies*.

